This article has been retracted.

# Effect of Hierarchical Nursing Management in Patients with Hypertension Complicated with Cardiovascular and Cerebrovascular Risk Factors

**DOI:** 10.1155/2021/1246566

**Published:** 2021-11-29

**Authors:** Lu Dai

**Affiliations:** The Cardiovascular Medicine Department of the First Affiliated Hospital of Chongqing Medical University, Chongqing 400016, China

## Abstract

Hierarchical management is an essential component of nurse post management and an unavoidable tendency in nursing education. According to their existing condition, various hospitals around the country have actively tested the hierarchical usage and management model of clinical nurses, with some success. The application impact of hierarchical nursing care in patients with hypertension complicated by cardiovascular and cerebrovascular risk factors is the focus of this research. In a hospital, 300 patients with hypertension complicated by cardiovascular and cerebrovascular risk factors were chosen. All patients were split into two groups using the coin-throwing random method: the observation group received hierarchical nurse management and the control group received regular nursing management, with 150 cases in each group. The two groups' blood pressure, blood lipids, blood glucose, poor habits, rehospitalization rate, and cardiovascular and cerebrovascular problems were also examined. At the same time, the patients' poor mood and quality of life were assessed before and after the intervention. In the control group followed up for 1 year, the blood pressure compliance rate was 44.88%, the blood lipid compliance rate was 28.65%, the blood glucose compliance rate was 45.00%, the smokers with bad lifestyle habits were 26.57%, the overweight and obese were 23.5%, the high sodium was 31.67%, the rehospitalization rate was 15.48%, and the incidence of cardiovascular and cerebrovascular complications was 43.00%. The observation group's blood pressure, blood lipids, and blood sugar compliance rates rose substantially (*P* = 0.05) as compared to the control group. The occurrence of poor luck living habits, the rate of rehospitalization, and the incidence of cardiovascular and cerebrovascular complications were significantly reduced (*P* < 0.05). Before nursing intervention, there was no significant difference in the bad mood scores SAS, SDS, and quality of life between the two groups of patients (*P* > 0.05); after nursing intervention, compared with the control group, the observation group's bad mood scores were significantly reduced, physical factors, psychological factors, and total scores all increased significantly, and the difference was statistically significant (*P* < 0.05).

## 1. Introduction

With the advancement of the social economy, people's living standards and modes are gradually changing, resulting in an annual increase in the incidence rate of hypertension, a prevalent chronic condition [1]. Hypertension is also often linked to cerebrovascular diseases, heart failure, and other cardiovascular and cerebrovascular complications, all of which can endanger patients' lives and impose a tremendous psychological and financial strain on their families. Hypertension is a systemic illness, according to studies, and its etiology is linked to a number of risk factors, including polygenic inheritance and the environment [2]. When the illness is coupled with other risk factors including diabetes, hyperlipidemia, and smoking, the risk of complications, rehospitalization, and possibly death increases [3]. Effective and scientific nursing interventions can help patients' prognoses by reducing the incidence of risk factors. As a result, one of the hotspots has been the investigation of efficient nursing approaches [4].

Hierarchical management is primarily concerned with integrating and allocating resources according to the position and professional ability of nurses, as well as implementing scientific management at various levels, in order to maximize the utilization of nursing resources and give better play to the nursing level of nurses [5]. Nursing human resource management is the process of arranging and effectively utilizing nursing staff in accordance with certain standards and norms in order to maximize people's abilities, fully stimulate personal potential, mobilize nursing staff's work enthusiasm, improve nursing work efficiency, and achieve organizational goals [6]. Many nations across the globe have now separated nursing personnel into various levels with clearly defined post responsibilities at all levels [7]. O'Grady [8], a human resource management technique for molding the working capacity of nursing staff at various levels according to a set of criteria, developed the concept of “level specific ability” in 2000. Since the 1950s, nations such as the United States and the United Kingdom have used a nurse rating system to assign nursing duties based on grades in order to better manage nursing human resources. In 2007, Almeida et al. [9] stated that hierarchical nursing management is a standardized and target management split into distinct levels and levels based on the position, professional title, and professional competence of nurses. Nurses preside over or take care of a certain job according to a given level or level, each in his or her own position, fulfill his or her own duties and obligations, and achieve unified management in strict accordance with organizational rules [10].

According to the requirements of nurses' position, professional title, and professional competence, the hierarchical usage of nurses is separated into distinct levels and different degrees of standardized management and target management [11]. Nurses are classified into five categories in the United States, based on their education and work experience, including nurse management (nm), nurse practitioner (NP), registered nurse, licensed practical nurse (LPN), and certified nursing assistant (CNA). A, B, and C nurses; D; class E registered nurse; F-level nurses with more seniority; G; H-level experienced senior nurse; and level I ward manager are the nine classes of British nurses. Registered nurses (RN), assistant nurses (EN), and nurses (N) are the three levels of nursing in Singapore (HCA). The number of nurses has risen substantially in recent years as a result of extensive advertising of high-quality nursing services [12]. Certain hospitals, based on their present circumstances, continue to actively investigate the implementation techniques of hierarchical nursing management, actively attempt the hierarchical use and management mode of clinical nurses, and have achieved some successes, primarily in five areas: increasing the quality of nursing care and the work happiness of nurses Patients' happiness, physicians' satisfaction with nurses' performance, and nurses' academic competence all improved [13]. However, there is currently no uniform hierarchical organisational structure framework or definition of nurses at all levels, and there is no accepted foundation for the hierarchical arrangement of nurses. [14]. Different researchers have different hierarchical settings of nurses, resulting in the diversification of hierarchical settings and names [15].

In some studies, nurses were employed according to their professional titles, and in others, nurses were stratified according to their professional titles, educational backgrounds, and ability levels [16]. Some are mainly based on the professional title, working years, and comprehensive ability of nurses, with reference to educational background, age, and other factors, although the stratification of nurses in each hospital is not the same [17]. However, the stratification basis of nurses in most hospitals includes factors such as nurses' actual working ability, professional title, clinical nursing working years, and educational background. This study introduced hierarchical nursing management into the nursing of patients with hypertension complicated by cardiovascular and cerebrovascular risk factors by searching the relevant cutting-edge knowledge of the literature database, combined with the reality of our department, in order to explore effective nursing measures and methods [18].

## 2. Related Work

The application of nurse hierarchical management model has been carried out in clinic. Kent et al. [19] obtained through the Delphi research that the actual working ability is the most key index to divide the nurse level, and the stratification of the actual working ability is also known as the stratification and advancement of the professional ability. Owen et al. [20] pointed out that in the establishment of advanced ability, the coordination between ability indicators and specialty standards should be considered. It can be seen that the ability standards at all levels should fully consider the characteristics of specialty. Norris et al. [21] set the nursing staff in ICU as head nurse, team leader, and responsible nurse according to different professional titles, education, and working ability and defines and strengthens the post responsibilities of personnel at all levels. Pien et al. [22] established a nursing staff organization and operation system based on the framework of “head nurse - responsible team leader - responsible nurse - auxiliary nurse” in the Department of Oncology. McGlothlin and Viele [23] divided the clinical nursing posts into “four level posts and three-level nurses” based on the professional title, educational background, seniority, specialized nursing ability, and other factors of nurses in neurosurgical wards, defined the corresponding working ability and requirements for nurses at all levels, and achieved good results. However, the application of nurse hierarchical management model in orthopaedic wards is rarely reported. Van Hecke is a fictional character. Van Hecke et al. [24] implemented the group work system in the orthopaedic department of Zhengzhou University's First Affiliated Hospital, dividing the nurses in the orthopaedic ward into four levels (responsible team leader, temporary team leader, responsible nurse, and mobile nurse), stipulating the job conditions and responsibilities of nurses at all levels, and linking each level to the bonus distribution. Through the implementation of nurse hierarchical management, patient satisfaction, health education coverage, nurse satisfaction, and pain control satisfaction were improved compared with those before the implementation, and the difference was statistically significant [25]. However, the study lacked the basis of nurse hierarchical framework, and the working conditions were stratified only according to education, working years, and professional titles, without considering the important index of working ability [26]. Therefore, the hierarchical management of nurses in orthopaedic ward needs to be further studied. According to the educational background, professional title, and evaluation of nurses, Zhao and Xia [27] divided the level of nurses into five levels: head nurse, specialist nurse, senior responsible nurse, primary responsible nurse, and assistant nurse; Fu et al. [28] divided nurses into four levels according to the qualification status of in-service nurses and the hierarchical principle of “ability first, conducive to work, personal development, and team construction,” stipulated the qualification of nurses at all levels, and implemented hierarchical training and assessment for nurses at all levels. In the practice of hierarchical management of nurses, Park and Choi [29] divided nurses into four levels, namely specialist nurses, senior responsible nurses, primary responsible nurses, and assistant nurses. Specialist nurses are under the management of the head nurse of the department and are arranged separately. In addition to completing the specialist nursing work in the undergraduate room, they also undertake the nursing guidance of the corresponding specialties in each ward of the hospital. The responsibilities of specialist nurses are as follows: participate in the nursing work of critical patients, focus on solving the specialist nursing problems of critical patients, and guide subordinate nurses; carry out nursing ward rounds, especially for critical patients; organize the formulation of nursing guidelines, nursing work standards, nursing quality evaluation standards, etc.; do a good job in health education for patients and their families and training for nurses; and set up specialized nursing clinics.

Friman et al.'s [30] research divides nurses into five levels. The hospital sets up a special committee to review the advanced points of nurses, designs an advanced point system, including the points of continuing education and work performance, and stipulates the minimum points for the advanced points of nurses at each level. Chang et al. [31] investigated the competence and advanced requirements at each level, combining clinical advanced with job performance assessment. According to Benner's seven dimensions of nursing practice, namely, help role, diagnosis and monitoring function, education/teaching function, management and monitoring of treatment intervention and course of treatment, quality monitoring, organization and coordination, and emergency response, they describe the core competencies that nurses should have in this dimension. Each dimension has three performance levels: need to develop, meet the standard, and exceed the standard. Karlsson et al. [32] think that a clinical ladder programme is important because it may offer nurses with professional growth opportunities and can be utilized as an incentive mechanism for nurses, all of which contribute to strengthening the stability of the nursing team. The initiative was extensively utilized as a successful strategy to minimize the loss of nurses in the 1980s, when there was a scarcity of nurses. The project mostly adopts Benner's model from novice to expert. According to clinical ability and work performance, nurses are divided into five levels: novice, senior novice, competent, proficient, and expert. When carrying out clinical advanced projects, some hospitals are stratified according to different fields of nursing specialty. For example, the nurse level of tempo general hospital has three fields and four levels. N1 is a probationary period. Generally, it can enter N2 after 6 months of practice. After that, there are three development channels, namely clinical, management, and education. N3 of the management channel is the assistant head nurse, and N4 is the head nurse; N3 of the clinical channel is the clinical nurse, and N4 is the clinical nursing expert.

## 3. Data and Methods

### 3.1. Specific Route

The main research steps are to establish the basic framework of hierarchical classification and four standards of nursing staff, form the first round of questionnaire and questionnaire cycle, and establish the hierarchical classification of nursing staff and four standards of each level. The expert prediction team is responsible for the specific organization and management of each stage. Six experts in nursing clinical management, nursing administration, nursing education, and nursing education management comprise the expert prediction team. The technical route of the study is shown in Figure 1.

### 3.2. General Information

300 patients with hypertension complicated with cardiovascular and cerebrovascular risk factors treated in our department were included in this project. According to the principle of clinical prospective research and the coin-throwing random method, all patients were divided into two groups, that is, the observation group was given hierarchical nursing management mode and the control group was given routine nursing management mode, with 150 cases in each group. The research plan of the project shall be implemented after being approved by the ethics committee of our hospital. There was no significant difference in the basic condition of the 2 groups between the 2 groups, such as gender, smoking history, drinking history, hypertension history, diabetes history, education level, age, and duration of disease. There was no significant difference between the 2 groups (*P* > 0.05) (see Figure 2).

### 3.3. Inclusion and Exclusion Criteria

Inclusion criteria are as follows: “hypertension-” related diagnostic criteria: (1) age: 18~75 years; (2) those who meet the diagnostic criteria and have at least one of smoking, dyslipidemia, impaired glucose tolerance (or impaired fasting glucose), and overweight or obesity (body mass BMI higher than 24 kg/m^2^); and (3) those who have normal cognitive function, can communicate normally, and signed informed consent. Exclusion criteria are as follows: (1) patients with other serious physical diseases and important organ failure; (2) patients with mental illness; and (3) pregnant and lactating women.

### 3.4. Nursing Management Measures

The control group received routine nursing management, which meant that the department's head nurse assigned work based on the nurses' individual characteristics and nursing experience, defined and divided nursing staff responsibilities, created requirements and work arrangements based on their responsibilities, and implemented a reward and punishment system. Observation group is as follows: a hierarchical nursing management mode was adopted, as follows: (1) firstly, the nursing staff of our department were divided into N1-5 different levels according to their educational background, working years, and professional titles, and different job responsibilities were given according to their levels, as shown in Figure 3. (2) Secondly, according to the seven steps of risk integration management in the patient safety guide, we formulate the eight-step APRDAPIE procedure intervention process, namely, evaluation (A), identification (R), report (R), confirmation (D), analysis (A), plan (P), implementation (I), and evaluation (E). Specifically, from the beginning of admission, the responsible nurse shall evaluate the patient's eating habits, living habits, medication, etc. (A) Once it is identified (R) that the patient already exists or has potential risks, the responsible team leader shall be informed in time for reevaluation, confirmation (D) and analysis (A). Generally, the nursing plan (P) for the patient shall be formulated within 24 hours, communicate with the patient's family members, patients, and responsible nurses to confirm the smooth implementation of the nursing plan (I), and give timely guidance in the implementation process. The responsible team leader shall regularly evaluate the nursing effect (E) and revise the nursing plan according to the evaluation results, until the nursing effect is achieved. (3) Nursing plan is as follows: it mainly includes five aspects: health education, establishment of hypertension risk factor management file, behavior intervention, observation of adverse reactions, and follow-up. Health education is primarily focused on gaining a thorough understanding of the prevalence of hypertension in order to emphasise the significance of food, tobacco, and alcohol in the prevention and treatment of hypertension as well as cardiovascular and cerebrovascular risk factors. It can be carried out orally or in the form of hanging health knowledge cards in front of the bed according to the patient's situation, and the responsible team leader will carry out the basic information of the patient, collect and manage the files including risk factor assessment and monitoring results, detect the drug reaction of patients, and timely inform the competent doctor for treatment. We intervene the patients' bad living habits, medication compliance, and other behaviors, sort them according to different risk factors of different patients, achieve the intervention objectives step by step, and start the follow-up after the patients are discharged from the hospital. The time is 1 week and 1 month after discharge and can be reduced to once every 3 months after three months. The follow-up is conducted in the form of telephone follow-up for 1 year, to follow up the blood pressure, cardiovascular and cerebrovascular risk factors, and complications of patients, and make records for reference.

## 4. Results and Analysis

### 4.1. Comparison of Blood Pressure Compliance during 1-Year Follow-Up

After one year of follow-up, there was no loss of follow-up in both groups. Compared with 44.88% in the control group, the blood pressure compliance rate in the observation group increased significantly (*P* < 0.05). It can be seen that the blood pressure of the observation group was well controlled, as shown in Figure 4.

### 4.2. Comparison of Cardiovascular and Cerebrovascular Risk Factors during 1-Year Follow-Up

Compared with the control group, the compliance rate of blood lipid and blood glucose for one year was 28.65%, 45.00%, and 26.57% of smokers, 23.5% of overweight and obese, and 31.67% of high sodium salt. Compared with the control group, the compliance rate of blood lipid and blood glucose in the observation group increased significantly (*P* < 0.05), and the incidence of bad living habits decreased significantly (*P* < 0.05). It can be seen that the improvement of cardiovascular risk factors such as blood lipid, blood glucose, and bad life in the observation group is better, as shown in Figure 5.

### 4.3. Comparison of Rehospitalization and Cardiovascular and Cerebrovascular Complications after 1-Year Follow-Up

The rehospitalization rate and the incidence of cardiovascular and cerebrovascular complications in the observation group were significantly lower than those in the control group (15.48% and 43.00%, *P* < 0.05). It can be seen that the rehospitalization and the incidence of cardiovascular and cerebrovascular complications in the observation group were reduced, as shown in Figure 6.

### 4.4. Comparison of the Improvement of Bad Mood between the Two Groups before and after Intervention

Before nursing intervention, there was no significant difference in SAS and SDS between the two groups (*P* > 0.05); after nursing intervention, compared with the control group, the adverse emotion scores of patients in the observation group also decreased significantly, and the difference was statistically significant (*P* < 0.05). It can be seen that the nursing measures of the observation group can not only better improve the physical symptoms of patients but also significantly improve the bad mood, as shown in Figure 7.

## 5. Conclusion

The continuous development of hypertensive diseases can lead to high disability, recurrence, or even mortality in patients. The reasons are found not only related to blood pressure but also mainly due to its own risk factors. Studies have confirmed that dyslipidemia, smoking, obesity, high blood sugar, and other common cardiocerebrovascular risk factors for hypertension, such as nutritional intervention, behavioral therapy, and other active interventions, can better reduce the level of risk factors and the occurrence of adverse events. Weight management, especially for obese individuals, may help lower blood pressure, blood lipids, and blood sugar levels, resulting in a stronger preventative impact. Hierarchical care is the nursing measure derived from the different needs of patients under this situation. In order to better improve the quality of care, in this project, nursing staff are classified according to their academic qualifications, working years and professional titles, rational deployment of human resources, and differentiation of work responsibilities, to make the best use of people, and people do their own responsibilities, better cooperate with work, and coordinate in arranging nursing projects and formulating work processes in accordance with the ARRDDAPIE eight-step procedure, so as to realize a nursing team model with a clear division of labor, avoid problems such as unclear responsibilities in the previous nursing model, and formulate targeted nursing measures. The results showed that the blood pressure compliance rate of the control group for 1 year was 44.88%, the blood lipid compliance rate was 28.65%, the blood glucose compliance rate was 45.00%, the smokers in bad lifestyle habits were 26.57%, the overweight and obese 23.5%, and the high sodium 31.67%. The hospitalization rate was 15.48%, and the incidence of cardiovascular and cerebrovascular complications was 43.00%. The observation group's blood pressure, blood lipid, and blood glucose compliance rates rose substantially (*P* = 0.05) as compared to the control group. It is precisely because of the adoption of this nursing measure that not only targeted nursing can be carried out, but it is also conducive to the evaluation and correction of nursing effects, ensuring that patients receive personalised continuous nursing interventions, preventing patients from developing bad living habits, and requiring rehospitalization. Cardiovascular and cerebrovascular problems were substantially decreased (*P* = 0.05), which had a larger influence on the therapeutic effect.

With the growing extension of the definition of health, it has moved beyond physical health to psychophysical health, with a focus on mental health. In this process, the scope of nursing work has expanded accordingly. Nurses are no longer the simple executors of medical orders in the past but have expanded into consultants and educators. At the same time, it is undeniable that people's requirements for mental health are increasing day by day. The increase of anxiety and depression caused by diseases seriously affected the quality of life of patients, while hierarchical nursing management gave targeted nursing intervention measures according to the different conditions of patients. The results showed that before nursing intervention, there was no significant difference in SAS, SDS, and quality of life between the two groups (*P* > 0.05); after nursing intervention, compared with the control group, the scores of adverse emotions in the observation group decreased significantly, and the physical factors, psychological factors, and total scores increased significantly (*P* < 0.05).

In conclusion, hierarchical nursing management can better reduce the incidence of high-pressure complicated with cardiovascular and cerebrovascular risk factors, reduce the incidence of complications, improve patients' bad mood, and improve their quality of life. However, due to the limited research time and energy, there are some problems in this study, which need to be improved, such as the comparison of the compliance rate of blood pressure in different groups, and the confirmatory study to further expand the sample size.

## Figures and Tables

**Figure 1:** Research technology roadmap.

**Figure 2:** Comparison of basic conditions between the two groups.

**Figure 3:** Hierarchical nursing management of nurses.

**Figure 4:** Blood pressure compliance in 1 year of follow-up.

**Figure 5:** Comparison of cardiovascular and cerebrovascular risk factors during one-year follow-up.

**Figure 6:** Comparison of rehospitalization and cardiovascular and cerebrovascular complications after 1-year follow-up.

**Figure 7:** Comparison of adverse mood improvement between the two groups before and after intervention.

## Data Availability

The data used to support the findings of this study are included within the article.
